# Analyzing trends in the spatial-temporal visitation patterns of mainland Chinese tourists in Sabah, Malaysia based on Weibo social big data^☆^

This article has been retracted.

**DOI:** 10.1016/j.heliyon.2023.e15526

**Published:** 2023-04-19

**Authors:** Rayner Alfred, Zhu Chen, Oliver Valentine Eboy, Zhang Luxuan, Li Renjie

**Affiliations:** a Creative Advanced Machine Intelligence Research Centre, Faculty of Computing and Informatics, Universiti Malaysia Sabah, Jalan UMS, 88400 Kota Kinabalu, Sabah, Malaysia; b Faculty of Social Sciences and Humanities, Universiti Malaysia Sabah, Jalan UMS, 88400 Kota Kinabalu, Sabah, Malaysia; c Faculty of Engineering, Universiti Putra Malaysia, Malaysia; d Faculty of Geographical Sciences, Hebei Normal University, China

**Keywords:** Social big data, Spatial-temporal visitation pattern, Spatial overlay analysis, Chinese tourists

## Abstract

Conducting on-site surveys to assess tourists' spatial visitation patterns and preferences is both time and labor intensive. However, an assessment of regional visitation patterns based on social media data can be an important decision-making tool for tourism management. In this study, an assessment of the visitation patterns of Chinese mainland tourists in Sabah is conducted to identify high-visitation hotspots and their changes, as well as large-scale and small-scale temporal characteristics. The data is sourced from the Sina Weibo platform using web crawler technology. In this work, a spatial overlay analysis was used to identify the hotspots of Chinese tourists' visits and the spatial and temporal variations. The results of the study revealed that the hotspots visited by Chinese tourists prior to 2016 have shifted from the southeast coast of Sabah, to the west coast of Sabah. At a small scale, Chinese tourists' visitation hotspots were mainly concentrated in the urban area along the southwest coast of Kota Kinabalu, shifting to the southeast of the urban area in 2018. This study provides insights into the applicability of social media big data in regional tourism management and its potential to enhance fieldwork.

## 1 Introduction

The development of Internet technology and social media has brought about tremendous changes in the tourism industry [1], [2], [3], [4]. Tourists can use social media for guidance or useful information before or during their trip [5], [6]. But before the spread of internet technology (e.g., cloud computing [7]) and social media, this information was mainly obtained through public institutions, travel books or resources [8]. Social media shows good interactivity and timeliness, making users more willing to share their lives on social media platforms [9], [10]. This also makes social media the main carrier of the digital media era and has been widely recognized and supported by the society [11], [12].

The information shared by users on social media platforms generates large-scale structured and unstructured data, which form big data and usher in the era of big data [13], [14], [15]. The information released by tourists on social media platforms can reflect the attention and visits of tourists to tourist destinations. The attention and visit volume of tourists will affect the management elements of the tourist destination, such as the supporting facilities (e.g., hotels, restaurants, entertainment) and future planning of the tourist destination. In addition, the economic benefits brought by the increase in the number of tourist visits ensure the stability of the development and protection of the tourist destination, thus improving the management capability of the tourist destination [16], [17]. Therefore, there is a need to assess the spatial visitation patterns and tourists characteristics of tourism destinations in order to obtain useful lessons in tourism management.

The identification of visitor spatial access patterns and the assessment of tourist destinations are usually based on interviews or questionnaire assessments, and different participants are considered in the process [18], [19]. However, the information collected through interviews or questionnaires is limited, and the temporal and spatial characteristics of tourists visiting multiple tourist destinations cannot be fully considered and reflected [20], [21]. Interviews, questionnaires, supporting analysis and geospatial analysis are representative methods of research to evaluate regional tourism and to quantify potential tourism destinations [22], [23]. But, collecting a large number of tourist information from different tourist destinations is time-consuming and expensive [24]. Therefore, such as tourists' preferences for different tourist destinations and the characteristics of visiting patterns within tourist destinations, these basic issues of public participation are difficult to determine, and it is necessary to explore the preferences and impressions of tourists visiting multiple tourist destinations.

About 2.5 exabytes of social media data are generated every day, through which the preferences and behaviors of different tourists can be mined, so social media big data is of great significance for evaluating tourist destinations [25], [26], [27]. Previous studies have determined that social media big data can reflect tourists' visiting trends to tourist destinations and can analyze tourists' different spatial visiting patterns and their relationship with tourism attributes [28], [29].

Some tourist destinations in developing countries have high recognition and conservation value, but the data quality of the relevant field data is poor [30], [31]. Nevertheless, the number of visits to tourist destinations and protected areas in developing countries has increased significantly [32], [33]. And developing countries mainly use field data to evaluate or inspect tourist destinations. Therefore, when using social media data to research and evaluate tourist destinations, it is necessary to consider the applicability and validity of social media data.

In 2019, about 3.1 million Chinese tourists visited Malaysia, making China the third-largest source market for international arrivals, based on Tourism Malaysia data. However, due to fears of another Covid-19 wave, several parties have called for the government not to allow entry for travellers from China [34]. In Sabah, tourism industry sector contributed 46.1% of the Sabah state annual revenue [35]. Thus, this research concentrated on Chinese tourists in Sabah, Malaysia.

There are no studies that have applied social media data to evaluate tourist visitation patterns in Sabah, Malaysia. Although the applicability and validity of data needs to be considered in applying social media data for tourism research, social media data can be a good remedy for the lack of survey data. The work of this research has been motivated by several studies that have shown the spatial–temporal-based big data can provide new insights gained from location-based social media data and understand human spatial–temporal behavior patterns [36], regulate and optimize tourism management services [37] and improve the quality of tourists using spatial–temporal [38], better understand human spatial–temporal behavior patterns and try to provide practical solutions to problems such as congestion and varying activity levels in tourism industry [39].

The aim of this study is to apply and validate a modeling method for mining key information about tourist destinations in Sabah, Malaysia using social media big data. Based on the aim of this research, here are three research questions that will be addressed in this work; 1) Is it feasible to collect the appropriate data on social media platforms and store in a geo-database? 2) What indicators of tourist interest are reflected and how these hotspots are distributed in space and time?

Thus, the objectives of this work are firstly, to investigate the best practice available to design and create a geo-database to store tourist data captured from social media platform, and then to adapt and implement the Kernel Density Analysis (KDA), Spatial Overlay Analysis (SOA) and Standard Deviation Ellipse Analysis (SDE) to visualize the tourist data and perform spatial analysis.

The contributions of this work include the findings related to the distribution of tourist destinations and related facilities in Sabah, Malaysia, and also the identification of high-traffic areas of Chinese tourists on both large and small scales.

Sabah, Malaysia is a famous tourist destination in Asia and even the world. Through Sina Weibo (http://www.weibo.com), we collected relevant information about Chinese tourists visiting Sabah, and explored the time and space visiting patterns of Chinese tourists. In addition, according to the time series, spatial overlay analysis is used to discover the preference characteristics of tourists in different periods. Finally, differences in existing tourist destinations and related facilities and spatial access patterns of tourists are analyzed. This study applies social media big data to provide new perspectives and insights into the application of Malaysian Sabah managers in tourism planning, development and management, while also including the effectiveness and limitations of their use. The findings are expected to help Sabah managers use social media big data to develop healthy and sustainable regional tourism destinations with limited field data.

## 2 Data and methods

### 2.1 Study area

Sabah is located in northern Borneo, between 115^∘^24' E to 118^∘^48' E and 4^∘^12' N to 6^∘^30' N, and is a state in Malaysia. Sabah has a total land area of nearly 74,500 square kilometers and a total coastline of 1,743 kilometers [40]. As Sabah's coastline faces three oceans, the region has extensive marine resources.

Sabah's coastline is rich in forest resources, mainly mangroves and Nipa forests. The coastal areas of Sabah's east and west coasts are dominated by beaches [41]. The terrain of the northern part of Sabah is dominated by mountains, the main mountain range being the Crocker Mountains. Mount Kinabalu is the highest mountain in the region with an elevation of approximately 4095 meters [42]. The Kinabatangan River is the second longest river in Malaysia and is located on the east coast of Sabah.

Sabah is famous for its beautiful natural scenery and cultural landscape, and is a famous tourist destination in Malaysia and even the world. Sabah is divided into 25 districts, of which Kota Kinabalu is the capital of Sabah. Apart from Kota Kinabalu, Sabah's major cities include Tawau, Sandakan, and Semporna. As shown in Fig. 1. In addition to Sabah's 25 districts and cities, it also includes surrounding islands and the Federal Territory of Labuan.

**Figure 1:** Overview of Sabah, Malaysia.

### 2.2 Data source

Since this work studies the Chinese tourists' visitation patterns in Sabah, Weibo data will be used as this is the major search engine that is mostly used in China.

#### 2.2.1 Data collection and validation

In 2009, Sina launched the Chinese micro-blogging site Sina Weibo, the first and most popular social media platform in China [43] and is publicly accessible to users. Using the written web crawler program, the target data can be easily collected from the Sina Weibo platform to automatically obtain web page data [44], [45]. Due to the limited interface provided by the Sina platform to developers, this study uses the place/nearby_timeline interface officially provided by Sina to collect data in chronological order, that is, the Weibo platform collects data once a month. However, in the collected text data, many Weibo posts were not posted by Chinese tourists visiting Sabah but were irrelevant information such as marketing and recruitment posted by travel agencies or advertisers. These data undoubtedly have an impact on the accuracy of subsequent analysis results. Therefore, to avoid the impact of these data on the accuracy of the analysis results, such data needs to be eliminated. The content of this type of data has more obvious keywords, such as recruitment, agency, company, promotion, etc. By summarizing these keywords and constructing a dictionary to match the text content in the data, data posted by users who are obviously not tourists in the data are eliminated. In the end, after preliminary data analysis of Weibo, from April 2014 to July 2019, a total of 100,365 Weibo entries were collected, after removing the irrelevant data.

Property location data in Sabah is mainly provided by OpenStreetMap (http://www.openstreetmap.org). OpenStreetMap provides a variety of ways for users to download map resources, where the geographic information is provided voluntarily and contains accurate spatial data for users to use [46]. Sabah's main tourist destinations and tourism supporting settings are obtained in point files or polygon files, including natural attractions, cultural attractions, and tourism-related supporting settings (e.g., hotels, restaurants, entertainment, etc.)

In order to verify the rationality of the number of Weibo as a proxy indicator of tourists, the number of Chinese tourists entering Sabah and the number of Weibo were compared. The number of international tourist arrivals in Sabah reflects the activity of tourists from various countries visiting Sabah, Malaysia. The collected Weibo data was from April 2014 to July 2019, and the whole year of Weibo data was selected for statistical summary on a monthly basis, from January, 2015 to December, 2018. Correspondingly, the number of inbound Chinese tourists visiting Sabah is counted on a monthly basis. Therefore, a total of 48 datasets are included, excluding the number of Weibo in 2014 and 2019, the number of Weibo from 2015 to 2018 is compared with the corresponding number of Chinese tourist arrivals on a monthly basis. There are 64 months of aggregated data (Nmax) generated according to the timestamp from April 2014 to July 2019. However, only 48 months (N) will be used (data aggregated monthly for year 2015 to 2018) out of 64 months to verify the number of microblogs that reflect the number or inbound Chinese tourists in Sabah.

### 2.3 Methods

Previous scholars that have conducted studies related to spatial-temporal analysis of tourists include investigating the spatial associations of urban tourism phenomena by using GIS and statistical methods to examine the relationships between hotels and land use types, attractions, transportation facilities, and the economic variables of the tertiary planning units in which the hotels are located [47], exploring the spatial pattern of China's tourism efficiency and the spatial heterogeneity of the influencing factors in depth [48], exploring the spatial-temporal features of ancient village tourism over three important time nodes of rural tourism development (in Zhejiang, China), as well as the contributing factors at both the provincial and prefectural city levels by using the geographic information system (GIS) spatial analysis method and the exploratory spatial data analysis model [49], investigating the impact of spatial-temporal variation on tourist destination resident quality of life [50], investigating the tourists' spatial-temporal behavior patterns based on GIS visualization and clustering methods from a microscopic perspective [51] and investigating intra-attraction tourist spatial-temporal behavior patterns using the concept of the space–time path of time geography [52].

In contrast, in this work, three methods are combined to analyze visitation patterns in Sabah based on Weibo Social Big Data to determine the spatial and temporal distribution of the visitor's area of interest, to identify high-traffic areas of Chinese tourists on both large and small scales, and to study the equilibrium degree of regional spatial distribution of tourist destinations in Sabah. These methods are Spatial Overlay Analysis (SOA) [53], Kernel density analysis (KDA) [54] and Standard Deviation Ellipse Analysis (SDE) [55]. SOA is accomplished by joining and viewing together separate data sets that share all or part of the same area. Thus, SOA is best used to determine the spatial and temporal distribution of the visitor's area of interest. KDA calculates the density of point features around each output raster cell and therefore it is best used to study the areas where Sabah tourist destinations gather to form larger tourist destinations. KDA is very much like histograms, but have two significant advantages. 1) Information isn't lost by “binning” as is in histograms, this means KDEs are unique for a given bandwidth and kernel. 2) They are smoother, which is easier for feeding back into a computer for further calculations. Finally, SDE is often used to describe the direction distribution of geographic features and is one of the commonly used methods in geostatistical analysis. Thus, SDE is best used to study the equilibrium degree of regional spatial distribution of tourist destinations in Sabah. Fig. 2 illustrates the flow chart of activities carried out in this work.

**Figure 2:** Flow chart of activities for Spatial-Temporal Analysis of Visitation Patterns in Sabah.

#### 2.3.1 Identifying the spatial-temporal visitation pattern of tourists

In this study, the collected Weibo data has precise location coordinates, so the number of Weibo is used as an indicator to identify tourists' spatial-temporal visiting patterns. The number of Weibo is considered here as a surrogate indicator of tourists.

At different spatial scales, the number of Weibo is calculated according to grids of different areas. On a large scale, the number of Weibo is calculated according to a grid of 11 km × 11 km. On a small scale, the number of Weibo is calculated according to a grid of 1 km × 1 km. The collected Weibo data was visualized using ArcGIS software based on the location information in the data. Sabah, Malaysia is divided into 1400 grids according to a grid of 11 km × 11 km. Kota Kinabalu is divided into 928 grids according to a grid of 1 km × 1 km.

#### 2.3.2 Determining the spatial and temporal distribution of visitors' areas of interest using spatial overlay analysis (SOA)

Tourists' visiting preference features are mined and analyzed through spatial overlay analysis by using ArcGIS 10.2. The distribution of natural attractions, cultural attractions and tourism-related facilities in Sabah, using the kernel density to mine the spatial distribution pattern of tourist destinations. Differences in tourist spatial access patterns and the distribution of tourist destinations and related settings are revealed by standard deviation ellipse analysis.

In GIS, it is often necessary to extract spatial implicit information to obtain more valuable information. Superposition analysis is one of the common methods to extract spatial implicit information. Unlike location queries, overlay analysis generates new layers, and with overlay analysis, some features in the input layer are split by the boundaries of features in the overlay layer [56], [57]. The new layer generated by the overlay analysis contains the attribute information of the original two or more layer features. In addition, new spatial relationships are generated through overlay analysis, and attribute relationships of all layers are updated.

#### 2.3.3 Determining the magnitude of Sabah tourist destinations using kernel density analysis (KDA)

Kernel Density Analysis (KDA) uses a kernel function to calculate the size of each unit area of a point or line feature to fit each point or line to a smooth conical surface. Commonly used kernel functions include quadratic kernel function, normal kernel function and fourth-order polynomial kernel function [58]. In the kernel density analysis, the choice of the bandwidth *h* has a great influence on the results of the kernel density analysis. In applications, the value of the bandwidth *h* is flexible, and different bandwidths can be selected for testing to explore the smoothness of the estimated point-dense surface [59]. KDA can be used to calculate the density of features in a neighborhood around those features. For instances, KDA can be used to find the densities of houses, crime reports or density of roads or utility lines influencing a town or wildlife habitat.

#### 2.3.4 Investigating the equilibrium degree of regional spatial distribution of tourist destinations in Sabah using standard deviation ellipse analysis (SDE)

Standard Deviation Ellipse Analysis (SDE) is often used to describe the directional distribution of geographic features and is one of the commonly used methods in geostatistical analysis [60], [61]. Through this method, the distribution of elements can be displayed in the form of an ellipse, and the distribution direction of the elements is reflected by the long and short semi-axes of the standard deviation ellipse. The rotation angle represents the angle between the main axis and the true north direction after the axis of the element set is rotated clockwise by a certain angle.

## 3 Results

### 3.1 Distribution of tourist destinations and related facilities in Sabah

Due to the differences in socio-economic development level and natural geographical conditions in Sabah, Malaysia, the distribution of tourist destinations and related facilities in various regions is uneven. In order to more accurately and scientifically reveal the distribution of tourist destinations and related facilities in Sabah, Malaysia in different regions, the 25 cities in Sabah, Malaysia, the surrounding islands and the Federal Territory of Labuan are taken as regional geographical units. Destinations and facilities are listed in descending order, as shown in Table 1.

**Table 1:** Distribution of Tourist Destinations/Facilities in various regions of Sabah, Malaysia.

Name	# of Tourism Destinations /Facilities	Percentage of Tourism Destinations (%)	Cumulative proportion (%)
Kota Kinabalu	189	20.52	20.52
Sandakan	101	10.97	31.49
Sea Island	99	10.75	42.24
Kota Belud	67	7.27	49.51
Ranau	61	6.62	56.13
Papar	61	6.62	62.76
Labuan Federal Territory	58	6.3	69.06
Kinabatangan	40	4.34	73.40
Kudat	34	3.69	77.09
Tawau	31	3.37	80.46
Beluran	29	3.15	83.60
Lahad Datu	25	2.71	86.32
Tuaran	24	2.61	88.93
Keningau	16	1.74	90.66
Penampang	14	1.52	92.18
Beaufort	13	1.41	93.59
Kuala Penyu	11	1.19	94.79
Putatan	9	0.98	95.77
Kota Marudu	7	0.76	96.53
Nabawan/Pensiangan	7	0.76	97.29
Sipitang	5	0.54	97.83
Tenom	5	0.54	98.37
Semporna	5	0.54	98.91
Kunak	5	0.54	99.46
Tambunan	4	0.43	99.89
Tongod	1	0.11	100.00
Pitas	0	0	100.00
Total	921	100	

Fig. 3 shows a kernel density analysis of the Sabah tourist destinations and related facilities, with a bandwidth taken as 10,000 m. It can be seen from Table 1 and Fig. 3 that the distribution of tourist destinations and related facilities in Sabah, Malaysia is low in balance. Its tourist destinations and related facilities are mainly concentrated in Kota Kinabalu, Sandakan, the surrounding islands of Sabah area, Kota Belud, Ranau, Papar, the number of which are 189, 101, 99, 67, 61, 61 respectively, accounting for 62.76% of the tourist destinations in the entire Sabah area. Semporna, Kunak, Tambunan, Tongod, and Pitas have fewer tourist destinations.

**Figure 3:** The kernel density analysis of tourist destinations and related facilities in Sabah.

### 3.2 The applicability of social media big data in exploring tourists' spatial visitation patterns

By comparing the statistics of the arrival of international tourists from Sabah, Malaysia with the number of Weibo collected, it is verified whether the number of Weibo reflects the number of Chinese tourists visiting Sabah, Malaysia. The number of Chinese tourist arrivals among them is counted and summarized on a monthly basis. The collected Weibo data is from March 2014 to July 2019, and the entire year of Weibo data is selected for statistics and aggregation on a monthly basis, which are 2015, 2016, 2017, and 2018 respectively. Pearson correlation analysis of the number of Chinese tourists visiting Sabah and Weibo data using SPSS software, the following results are obtained.

Table 2 shows the results of descriptive statistics. As seen in Table 2, the maximum number of Chinese tourists visiting Sabah from January 2015 to December 2018 was 65,292, the minimum was 14,024, the mean was 34,302.3, and the standard deviation was 11,861.9. The maximum number of Weibo during this period was 4,427, the minimum was 81, the mean was 1,574.7, and the standard deviation was 1292.4, where *N* is the sample size.

**Table 2:** Descriptive statistics of Chinese tourists visiting Sabah and the number of Weibo.

Item	N	Min Value	Max Value	Mean	Std Dev
Chinese tourists visiting Sabah	48	14024	65292	34302.3	11861.9
The number of Weibo	48	81	4427	1574.7	1292.4

The correlation between the number of Chinese tourists visiting Sabah and the number of Weibo was fitted by SPSS regression analysis, as shown in Fig. 4. The R-squared in Fig. 4 indicates the square of the correlation coefficient. The correlation coefficient between the number of Chinese tourists visiting Sabah and the number of Weibo was 0.637 (p-value < 0.01, N=48). A test of the critical value of the correlation coefficient showed a critical value of 0.368 (p-value < 0.01) at a sample size N of 48. Thus there is a significant positive correlation between the number of Chinese tourists visiting Sabah and the number of Weibo. This shows that the number of Chinese tourists visiting Sabah has an impact on the number of travel-related Weibo published by Chinese tourists on the Weibo platform, and there is a significant positive correlation. Therefore, the Weibo data on the Weibo platform can reflect the travel activities of Chinese tourists in Sabah, Malaysia.

**Figure 4:** Scatterplot between the number of Chinese tourists visiting Sabah and the number of Weibo.

### 3.3 Spatial-temporal visitation patterns of Sabah tourists destinations at multi-scale

Based on the social media big data of Sina Weibo, the number of Weibo accounts reveals the tourist destinations in Sabah visited by Chinese tourists (Fig. 5). Combining social media data from April 2014 to July 2019, Kota Kinabalu and Semporna were the most frequently visited areas by Chinese tourists. In addition, time stamps are also used to show the changes in the density of tourists visiting the tourist destination at different times, as shown in Fig. 6. The results show that between April 2014 and December 2015, the largest number of Chinese tourists visited eastern Semporna, southern Tawau, and northeastern Sandakan. After 2016, the number of tourists visiting Kota Kinabalu and surrounding areas has increased significantly, becoming Sabah's most visited area by Chinese tourists. The number of Chinese tourist arrivals in southern Tawau and northeastern Sandakan has decreased significantly compared to before 2016. South Kota Belud and Pulau Mantanani Besar show areas with high Chinese tourist visiting.

**Figure 5:** Excavation of Visitation Patterns in Sabah Tourist Destinations.

**Figure 6:** Excavation of Visitation Patterns in Sabah Tourist Destinations from April 2014 to July 2019.

Small-scale social media data mining can help reveal the preferences and changes of tourist visiting patterns within tourist destinations. As the capital of Sabah, Kota Kinabalu is an important hub for international tourists visiting Sabah. And on a grand scale, Kota Kinabalu is also a hot spot for Chinese tourists to visit. After 2016, the number of Chinese tourists visiting Kota Kinabalu and surrounding areas has increased significantly, as shown in Fig. 7. In addition, changes in visiting patterns and preferences of Chinese tourists within the Kota Kinabalu region from 2016 to July 2019 were also visualized, as shown in Fig. 8. The results showed that the southwest of Kota Kinabalu was identified as a place frequently visited by Chinese tourists. Moreover, from 2016 to July 2019, the number of visits by Chinese tourists in the southwest region of Kota Kinabalu also showed differences. During 2016 and 2017, the most frequently visited areas by Chinese tourists were concentrated along the southwest coast of Kota Kinabalu. After 2018, the places most visited by Chinese tourists began to shift eastward.

**Figure 7:** Excavation of Visitation Patterns in Kota Kinabalu Tourist Destinations.

**Figure 8:** Excavation of Visitation Patterns in Kota Kinabalu Tourist Destinations from 2016 to July 2019.

In this study, Weibo-based spatial visitation patterns of Chinese tourists are matched with local knowledge of visiting hotspots. Semporna is a famous diving destination in Sabah, and both Pulau Mantanani Besar and Pulau Mantanani Besar have rich island tourism resources. South of Kota Belud is the location of Mount Kinabalu National Park. As the capital of Sabah, Kota Kinabalu not only includes abundant tourism resources, but also has convenient transportation conditions and sound tourism-related facilities. The city of Kota Kinabalu and the famous Tanjung Aru Beach are concentrated in the southwest area of Kota Kinabalu.

### 3.4 The association of Chinese tourists visitation patterns with Sabah's tourist destinations

The spatial distribution of tourist destinations in Sabah has some similarities to the preferences of Chinese tourists visiting Sabah, but also shows more significant differences. Standard deviation ellipse analysis can reveal more accurately the relationship between the spatial distribution of tourist destinations in Sabah and the visitation preferences of Chinese tourists.

The center of the spatial distribution of tourist sites and related facilities in Sabah is located at 116^∘^29'57.9'E, 5^∘^52'33.2'N. The center of the distribution of Chinese tourist visitation patterns is located at 116^∘^29'16.4'E, 5^∘^48'12.5'N (Fig. 9). The distance between the two is 8.14 km. From the rotation angle, the rotation angle of the ellipse of standard deviation of tourist places and related facilities in Sabah is 86.07^∘^, indicating that the distribution direction of tourist places and related facilities shows an east-west trend. The angle of rotation of the ellipse of standard deviation of Chinese tourist visitation pattern is 121.88^∘^, indicating a northwest-southeast trend in the direction of distribution of Chinese tourists. In addition, the spatial distribution direction of Chinese tourists' visits is more pronounced, but the distribution range is smaller, which also indicates a more concentrated area of Chinese tourists' visits.

**Figure 9:** Directional distribution of Sabah's tourist destinations and related facilities in relation to Chinese tourist visitation patterns.

In Fig. 10, at a small scale, the distribution center of tourist sites and related facilities in Kota Kinabalu is 116^∘^5'15.7'E, 5^∘^59'42.5'N. The distribution center of Chinese tourists in Kota Kinabalu is at 116^∘^3'57.3'E, 5^∘^58'11.4'N. The two distribution centers are 3.7 km apart. In terms of rotation, the standard deviation elliptical rotation angle of Kota Kinabalu tourist sites and related facilities is 55.15^∘^, and the standard deviation elliptical rotation angle of Chinese tourist distribution is 51.11^∘^. This indicates that both the spatial distribution pattern of Kota Kinabalu tourist destinations and the spatial distribution pattern of Chinese tourists' attention show a southwest-northeast trend. The direction of distribution of Kota Kinabalu tourist destinations and related facilities is more obvious from the long and short axes of the standard deviation ellipse. However, the distribution of Chinese tourists is smaller, with more pronounced centripetal force and more concentrated distribution.

**Figure 10:** Directional distribution of Kota Kinabalu tourist destinations and related facilities in relation to Chinese tourist visitation patterns.

Based on Figure 9, Figure 10, it can be concluded that at a small scale, Chinese tourists prefer to visit the main tourist attractions located at the main city. However, at a larger scale, most of the tourist attractions located near the Mount Kinabalu, Ranau, Penampang and Tambunan. These tourist attractions provide more nature-based facilities that involve and revolve around the area's natural products and will include either or all of the animals, plants and human cultural variety.

## 4 Discussion

### 4.1 Applicability of social media big data in assessing tourism

The combination of volunteered geographic information system and expert system can overcome the challenges in tourism management of different tourists visiting multiple destinations [62]. However, the application of such tools is time-consuming and labor-intensive. In contrast, data on social media platforms containing location information is effective in assessing tourist visitation patterns at scale. Using the location and time information on Weibo, this paper quantitatively analyzes the visiting patterns of Chinese tourists in various tourist destinations in Sabah. This model can also be used to analyze and compare tourists from different countries in Sabah and the tourism industry in a global context, as social media big data contains various spatial-temporal information of different tourists, which is cost-effective.

Although the application of social media big data in tourism requires a large amount of observational data to verify, the number of Chinese tourists visiting Sabah and the collected Weibo data are statistically significant (*r*=0.637, *p*=0.01). The analysis results show that social media big data can effectively identify tourists' visiting preferences and spatial differences in tourist hotspots.

In this study, the degree of tourists visitation to Sabah tourist destinations at different scales was mined and visualized. This information helps manage existing tourism activities as well as develop new tourism projects. It is also a new attempt to quantitatively evaluate cultural services in ASEAN countries and other countries. In addition, mining the visitation degree of different tourist destinations based on social media big data is crucial for the development of sustainable tourism [63]. The degree of visitation of the tourist destination can be used to further analyze the threatened area, such as the degree of tourists visiting more than its area carrying capacity.

In addition, the results of the standard deviation ellipse analysis show the association of Chinese tourist visitation hotspots with Sabah's tourist sites and related facilities. And there are significant differences at different scales. By further analyzing the textual content posted by tourists, the factors influencing tourists' visits can be further explored to develop targeted marketing strategies and tourism planning.

### 4.2 Effectiveness on regional tourism planning and management

Social media big data can support and assist managers and policy makers in regional tourism planning and tourism management. In this study, hotspots and visitation preferences of Chinese tourists in Sabah were identified. Differences in the spatial distribution of tourist visitation hotspots in relation to tourist destinations and related facilities were also identified.

For instance, it was found that the attention of Chinese tourists was mainly concentrated in coastal areas and islands. From April 2014 to the end of 2015, it was mainly concentrated in Semporna, Pulau Mantanani Besar, Sandakan and Tawau. After 2016, the attention of Chinese tourists was mainly concentrated in Kota Kinabalu, Semporna and Pulau Mantanani Besar. In addition, in the large-scale analysis of the relationship between the spatial distribution of Sabah tourist destinations and the spatial distribution of Chinese tourists' attention, it was found that there was no direct relationship between the spatial distribution of Sabah's tourist destinations and the spatial distribution of Chinese tourists' attention. Although the distribution centers of the two are similar, the south-eastern region of Sabah has attracted more attention from Chinese tourists and lacks fewer tourist destinations. On a small scale, it was found that Chinese tourists pay high attention to the urban area of Kota Kinabalu, the Chinese area near Damai Road and Tanjung Aru Beach. However, less attention was paid to the Kota Kinabalu City Mosque, Sabah University, Pulau Gaya and Tunku Abdul Rahman National Park near the city of Kota Kinabalu. From the study of the relationship between the spatial distribution of Kota Kinabalu tourist destinations and the spatial distribution of Chinese tourists' attention, it was found that the spatial distribution of Kota Kinabalu's tourist destinations and the attention of Chinese tourists show a certain correlation. The two show a certain similarity in terms of distribution center and distribution direction. However, it can be seen from this that Chinese tourists' attention to Kota Kinabalu's tourist destinations was concentrated in and around the urban area. Although there were more tourist destinations in the north-eastern area of Kota Kinabalu, their attention is relatively low.

This information can be used to develop or manage tourism activities [64], such as developing new tourism projects and related facilities along the southeast coast of Sabah, or developing new marketing models to direct tourists to the eastern coastal region of Sabah in order to increase the length of stay and regional tourism revenue. Managers can improve the quality and quantity of data by evaluating and managing the needs of different visitors through modern technology [21]. In this regard, social media data can be used to analyze and achieve deeper management goals, such as tourist satisfaction during the travel process, or changes in tourist visiting patterns before and after a particular event.

### 4.3 Coordination with sentiment analysis

Textual content in social media data can be a powerful tool for evaluating tourist satisfaction. Spatial visitation patterns do not fully represent tourists' sentiment or satisfaction with a destination, and sentiment analysis can help reveal the sentiment and distribution of tourists in a destination and further investigate the perceived value of tourists. This may help to understand the behavioral patterns of tourist visitation preferences, such as why Kota Kinabalu is the most frequently visited tourist destination by Chinese tourists. Combining sentiment analysis can reveal the diverse perceived values of tourists and also provide suggestions for tourism managers to improve services at the destination and increase tourist satisfaction.

## 5 Conclusion

This work firstly studied the realistic spatial pattern of Sabah tourist destinations, and on this basis, excavates the online attention of Chinese tourists at different spatial scales. In the end, the relationship between the spatial distribution of tourist destinations and the online attention of Chinese tourists at different scales is discussed.

This paper has proposed the application of social media data to identify the visitation patterns and preferences of mainland Chinese tourists in Sabah. The secondary objective is to also identify high-visit hotspots and their changes through the temporal attributes of social media data. Based on the findings obtained in this work, the Weibo dataset can be used to extract entities required to be stored in the geo-database. Furthermore, based on the data analysis conducted in this work, the following conclusions can be drawn related to the indicators of tourist interest and how these hotspots are distributed in space and time;

• The distribution of tourist destinations and related facilities in Sabah, Malaysia is uneven, mainly concentrated in Kota Kinabalu, Sandakan, the surrounding islands of Sabah area, Kota Belud, Ranau, Papar. Semporna, Kunak, Tambunan, Tongod, and Pitas have fewer tourist destinations and related facilities.
• The high-traffic areas of Chinese tourists on a large scale are in Kota Kinabalu and Semporna. Before 2016, Semporna, southern Tawau and northeastern Sandakan were the areas with the highest number of Chinese tourists; after 2016, Kota Kinabalu became the most visited area by Chinese tourists. South Kota Belud and Pulau Mantanani Besar are also frequently visited areas by Chinese tourists.
• On a small scale, the areas visited by Chinese tourists are mainly concentrated in the southwest of Kota Kinabalu (e.g., Ranau, Tambunan). Since 2016, the number of visits to the urban area of Kota Kinabalu has been decreasing year by year.

The association of tourist sites and related facilities with tourist visitation hotspots at different scales is also discussed. At large scales, Sabah tourist sites and related facilities show variability in terms of distribution direction, distribution extent, and distribution dispersion from tourist visitation hotspot areas. At small scales, tourist sites and related facilities in Kota Kinabalu show variability in terms of distribution range and dispersion of distribution.

In addition, this study also discusses the applicability of social media big data in the tourism industry. Although data from social media platforms is limited, this type of data is effective in mining and assessing tourism within an area. Through social media data, visitor visit patterns and preferences can be identified, and managers can develop policies to control visitor flow and behavioral changes. It is also an innovative tool for social media data to support destination management and the development of sustainable tourism. Finally, the field survey results combined with the advantages of social media data can provide managers with reliable information to promote the healthy and sustainable development of tourism in the region.

Data obtained from social media platforms may be biased. In addition, in different tourism activities, tourists' willingness to post content or photos is also different. For example, when tourists explore the island by speedboat, they may not like to take pictures in the process although they have a device connected to the Internet. The data quality of social media big data is affected by the GPS capabilities of tourists' mobile devices and internet access. Finally, there are differences in the access patterns shown by different social media platforms. Therefore, in future research, consider using social media big data from different platforms to mine tourists' visiting preferences and visiting degrees. In addition, this study collected 100,365 Weibo data from April 2014 to July 2019, which requires sufficient field data to verify the credibility of social media big data. Despite these limitations and obstacles, the findings of this study are still able to demonstrate the effectiveness of social media big data in mining tourists' visit preferences and degree of visit. The above issues still need further consideration and evaluation to improve the applicability of social media big data.

## CRediT authorship contribution statement

Rayner Alfred: Conceived and designed the experiments; Performed the experiments; Analyzed and interpreted the data; Contributed reagents, materials, analysis tools or data; Wrote the paper.

Zhu Chen: Conceived and designed the experiments; Performed the experiments; Analyzed and interpreted the data; Contributed reagents, materials, analysis tools or data; Wrote the paper.

Oliver Valentine Eboy: Analyzed and interpreted the data.

Zhang Luxuan: Performed the experiments.

Li Renjie: Contributed reagents, materials, analysis tools or data.

## Declaration of Competing Interest

The authors declare no conflict of interest.

## Data Availability

The authors do not have permission to share data.
